# Niacin protects against UVB radiation-induced apoptosis in cultured human skin keratinocytes

**DOI:** 10.3892/ijmm.2012.886

**Published:** 2012-01-12

**Authors:** FUQUAN LIN, WEN XU, CUIPING GUAN, MIAONI ZHOU, WEISONG HONG, LIFANG FU, DONGYIN LIU, AIE XU

**Affiliations:** Department of Dermatology, Third People’s Hospital of Hangzhou, Hangzhou 310009, P.R. China

**Keywords:** niacin, UVB, AKT, apoptosis

## Abstract

Niacin and its related derivatives have been shown to have effects on cellular activities. However, the molecular mechanism of its reduced immunosuppressive effects and photoprotective effects remains unclear. In this study, we investigated the molecular mechanism of the photoprotective effect of niacin in ultraviolet (UV)-irradiated human skin keratinocytes (HaCaT cells). We found that niacin effectively suppressed the UV-induced cell death and cell apoptosis of HaCaT cells. Existing data have shown that AKT activation is involved in the cell survival process. Yet, the potential mechanism of niacin in protection against UV-induced skin damage has thus far not fully been eluvidated. We observed that niacin pretreatment enhances UV induced activation of AKT (Ser473 phosphorylation) as well as that of the downstream signal mTOR (S6 and 4E-BP1 phosphorylation). The PI3K/AKT inhibitor, LY294002, and the mTOR inhibitor, rapamycin, largely neutralized the protective effects of niacin, suggesting that AKT and downstream signaling mTOR/S6 activation are necessary for the niacin-induced protective effects against UV-induced cell death and cell apoptosis. Collectively, our data suggest that niacin may be utilized to prevent UV-induced skin damage and provide a novel mechanism of its photoprotective effects against the UV radiation of sunlight by modulating both AKT and downstream mTOR signaling pathways.

## Introduction

Niacin has long been used in the treatment of high cholesterol, coronary heart disease, the skin disease Pellagra and age-related macular degeneration (AMD) (1,2). Niacin and its derivative, niacinamide, have been widely applied in skin care products, including moisturizers, anti-aging products, and rosacea treatments (3). It has been well-accepted that niacin has protective effects against skin photodamage induced by ultraviolet (UV)-radiation. A niacin derivative, myristyl nicotinate (MN), may enhance epidermal differentiation and barrier function in skin against photodamage, suggesting that niacin delivery may protect against UV skin damage and may be used in treating skin barrier impairment (4).

Niacin has the potential to influence cellular processes including DNA repair, genomic stability, the immune system, stress responses, signaling, transcription, apoptosis, metabolism, differentiation, chromatin structure and life span. In addition to its well-known redox functions in energy metabolism, niacin and its derivatives in the form of NAD and NADP, are required for the synthesis of cyclic ADP-ribose and NAADP, which are two major mediators of intracellular calcium signaling pathways (5).

A previous study (6) showed that niacin-deficient HaCaT cells with low NAD status develop a decreased growth rate due to an increase in apoptotic cells and an arrest in the G2/M cell cycle phase accompanied with accumulation of reactive oxygen species and increased DNA damage. This model of niacin deficiency has also allowed the identification of NAD-dependent signaling events critical in early skin carcinogenesis. Niacin deficiency in humans would cause sun sensitivity in the skin, indicative of deficiencies in responding to UV damage.

Furthermore, the identification of the nicotinic acid receptor in human skin keratinocytes provides a further link to niacin’s role as a potential skin cancer prevention agent and supports the role of the nicotinic acid receptor as a potential target for skin cancer prevention agents (7). While the exact mechanism through which niacin serves as a modulator agent for a critical resistance factor to prevent from UV-induced skin damage is still unknown. Cellular energy loss (8) and AMPK, AKT and eNOS activation (9) have been suggested as some of the niacin protective mechanisms.

UV is divided into UVC (200–280 nm), UVB (280–320 nm) and UVA (320–400 nm). UVB is of environmental significance, penetrating into the papillary area of the dermis and inducing DNA damages to the residing dendritic cells (DC)(10–12), as well as keratinocytes. These cells are perturbed both phenotypically and functionally, undergoing apoptosis upon UVB-radiation. Apoptosis can be induced in the region that suffers the greatest exposure and cells surrounding this area would also be partially damaged (10,12).

Apoptosis is the process of programmed cell death, which involves a series of morphological changes, including cell detachment, cell shrinkage, mitochondria leakage, chromatin condensation, and DNA fragmentation. This process is controlled by the balance between pro-apoptotic and anti-apoptotic signaling pathways (13). The PI3K/AKT and JNK phosphorylation cascades act as two important regulators, and will have an anti-apoptotic role in a variety of tissue culture models against stresses such as UV irradiation, matrix detachment, cell cycle disturbance, and DNA damages (14,15).

Previous studies in dendritic cells as well as keratinocytes have demonstrated that the cellular response to UV is composed of transactivation of cell surface growth factors, such as EGFR, and their downstream signal transduction machinery such as MAPK and PI3K/AKT (12,16–19). UV activates all three MAPK families including JNK, p38 and ERK in human keratinocytes and skin dendritic cells (12,20–25). While MAPK (JNK and p38) is responsible for UV-induced cell apoptosis, other cellular signals such as AKT serve as survival signals to fight against UV-induced widespread cell death (17,19,26,27). Activated AKT relays its survival signals in a number of ways including phosphorylation and inactivation of the pro-apoptotic BH3 protein BAD (28), members of the Forkhead family of transcription factors (29) and Mdm2, the negative regulator of p53 (30). However, the possible role of mTORC1 (mTOR complex 1), another important downstream target of AKT, in UV-induced cell death is not fully studied.

It is possible that niacin affects the cell status by protecting against UV-induced apoptosis and death. To determine the mechanism of niacin in HaCaT cells under UV, we measured the level of AKT and MAPK after UV irradiation. In this study, we demonstrate that UV radiation induces both AKT and MAPK activation. AKT and TSC2 are required for UV-induced mTOR/S6 activation (S6K and 4E-BP1 phosphorylation). Niacin pretreatment protects against UV-induced cell death and apoptosis in keratinocytes (HaCaT cells) by enhancing AKT/mTOR and S6 activation. Niacin may have a functional role in the pro-survival mechanism through activating the AKT/mTOR/S6 signaling pathway.

## Materials and methods

### Materials

Niacin (nicotinic acid) and DMSO were obtained from Sigma (St. Louis, MO, USA). Monoclonal mouse anti-β-actin, goat anti-rabbit IgG-HRP and goat anti-mouse IgG-HRP antibody were purchased from Santa Cruz Biotechnology, Inc. (Santa Cruz, CA, USA). The Annexin V-FITC kit was purchased from BD Biosciences (San Jose, CA, USA). The JC-1 probe cell apoptosis detection kit was provided by the Beyotime Institute of Biotechnology (Haimen, China). The p-EGFR (Tyr1068) antibody, and the p-AKT (Ser473), p-AKT (Thr308), p-S6K (Thr389), p-4E-BP1 (Ser65), p-S6 (S235/236), p-mTOR (Ser2448), p-p38 (Thr180/Tyr182), p-JNK(Thr183/Tyr185), p-ERK1/2 (Thr202/Tyr 204), and p-TSC2 (Ser 1462) antibodies, the AKT inhibitor LY294002, the mTOR inhibitor rapamycin, the Tuberin/TSC2 siRNA, and the p38 MAPK, JNK and the AKT1/2 antibodies were all from Cell Signaling Technology (Beverly, MA, USA). The EGFR inhibitor, PD153035 was purchased from Invitrogen (Carlsbad, CA, USA).

### Cell culture, transfection and UV treatment

The spontaneously immortalized human keratinocytes (HaCaT cell line) were cultured at 37°C in RPMI-1640 supplemented with 10% fetal bovine serum and 100 U/ml of penicillin/streptomycin as previously reported (31,32). The procedures for UV irradiation were similar to those described previously. For UV irradiation experiments, the cells were starved for 1 day and then washed twice with phosphate-buffered saline (PBS) before being exposed to UV irradiation using a germicidal lamp (emission wave, 290–320 nm; radiation intensity, 1.35 mW/cm^2^) SS-04B Sigma High-Tech Co., Ltd. (Shanghai, China). Doses of UV-irradiation were calibrated with a UVX radiometer also from Sigma High-Tech Co., Ltd. For siRNA transfection, cells were plated at a density of 3×10^6^ cells per 100-mm culture dish, incubated overnight, and then transfected with the indicated expression vectors, using Lipofectamine 2000 (Invitrogen, USA).

### Cell viability assay (MTT assay)

Cell viability was measured by the 3-[4,5-dimethylthylthiazol-2-yl]-2,5 diphenyl tetrazolium bromide (MTT) method (31). Briefly, cells were seeded in 96-well plates at a density of 1×10^4^ cells/well. Different seeding densities were optimized at the beginning of the experiments. After incubation for 24 h, cells were exposed to fresh medium containing reagents at 37°C. After incubation for up to 24 h, 10 μl of MTT tetrazolium salt (Sigma) dissolved in Hank’s balanced solution at a concentration of 5 mg/ml was added to each well and incubated in a CO_2_ incubator for 4 h. The DMSO (10 μl) was added to dissolve formazan crystals and then lysed on a shaker for 15 min. The absorbance value at 490 nm was measured with a microplate spectrophotometer (SoftMax^®^ Pro5, Molecular Devices, USA).

### Western blot analysis

As described previously (33), post treatment, cells were collected and lysed in RIPA buffer (10 mM NaPO_4_, pH 7.4/300 mM NaCl/0.1% SDS/1% Nonidet P-40/1% deoxycholic acid/2 mM EDTA) with protease inhibitors (Pierce, USA). Aliquots of 30–40 μg of protein from each sample (treated as indicated in the legends) were separated by 10% SDS-polyacrylamide gel electrophoresis (SDS-PAGE) and transferred onto a polyvinylidenedifluoride (PVDF) membrane (Millipore, Bedford, MA). After blocking with 5% BSA (Beyotime) for 1 h, membranes were incubated with specific antibodies overnight at 4°C followed by incubation with secondary antibodies (HRP-conjugated anti-rabbit or anti-mouse IgG at the appropriate dilutions) for 45 min to 1 h at room temperature. Immunoblotted membranes were developed using the ECL western blotting system (Thermo Scientific Biotechnology, USA). Quantification of appropriate bands on western blots was performed using the quantification software of the digital imaging system (ChemiDoc™ XRS^+^, Bio-Rad, USA).

### Confocal laser scanning microscope (CLSM)

As previously described (33), all cells were fixed with 4% formaldehyde in PBS for 30 min. Fixed cells were blocked with 10% BSA in PBS for 30 min at room temperature. Anti-p-AKT and anti-p-S6 polyclonal antibodies were used at 1 μg/100 μl in buffer (0.5% BSA in PBS) and incubated with the coverslip for 1 h. The antibodies were detected using appropriate secondary antibodies (goat anti-mouse or goat anti-rabbit; Beyotime, China) conjugated to Cy3 or FITC at 1:200. The processed slides were observed with a Confocal Laser Scanning Microscope (TCS SP2, Leica, Germany).

### Annexin V and propidium iodide (PI) staining

A cell apoptosis detection kit was used for Annexin V and PI staining. HaCaT cells were cultured in 35-mm dishes and were exposed to different treatments. Cells were harvested after up to 24 h incubation and washed in PBS twice. Cells were re-suspended in the binding buffer, and then the fluorescein-conjugated Annexin V and PI reagent were added to cell suspensions. After incubation in the dark for 15 min the percentage of apoptotic cells and necrotic cells were assessed by a flow cytometer (FACSCalibur, BD Biosciences, USA).

### Mitochondrial membrane potential assay

The JC-1 probe was used to measure mitochondrial depolarization. Briefly, cells were cultured in 6-well plates up to ~50% confluency, and after the indicated treatments cells were incubated with 1 ml of JC-1 staining solution (5 μg/ml) at 37°C for 20 min and rinsed twice with PBS. Mitochondrial membrane potentials were monitored by determining the relative amounts of dual emissions from mitochondrial JC-1 monomers or aggregates using an Olympus fluorescent microscope under Argon-ion 488 nm laser excitation. Mitochondrial depolarization is indicated by an increase in the green/red fluorescence intensity.

### Statistical analysis

The values in the figures are expressed as the means ± standard deviation (SD). All experiments were repeated at least three times. Experimental groups were compared by one-way ANOVA analysis of SPSS 16.0. Mean differences were considered significant (P<0.05) and highly significant (P<0.01).

## Results

### Niacin protects against UV-induced cell death and apoptosis in keratinocytes (HaCaT cells)

By using the cell viability MTT assay, first we investigated the possible protective effects of niacin against UV-induced cell death. As indicated in Fig. 1, cells were pretreated with a dose-dependent course of niacin (0, 5, 10, 20 and 40 μM), after with or without UV (30 mJ/cm^2^) as indicated in similar studies. There was no significant dosage effect with up to 40 μM of niacin in the control groups. As expected, UV treatment caused a marked decrease in cell viability. The viable cells dropped to 79.35±1.21% (n=4) of the control within 24 h of 30 mJ/cm^2^ UV radiation. In the presence of niacin, the cell viability was markedly recovered to 90.21±7.09% (P<0.01) at 20 μM of niacin in comparison to the UV-treated and niacin-free group. Signiflcant improvement of cell viability occurred with a graded increase in niacin concentrations from 5 to 20 μM, and showed a declining trend at 40 μM with UV treatment. Next we assessed whether niacin can inhibit UV-induced cell apoptosis. Data in Fig. 2C clearly demonstrate that 20 μM with niacin pretreatment diminishes UV induced cell apoptosis in HaCaT cells as evidenced by the Annexin V and PI staining assay (Fig. 3). Normal cells stained with the JC-1 probe emitted mitochondrial red fluorescence and limited green fluorescence. Aggregated JC-1 has a high mitochondrial membrane potential and emits red fluorescence but will turn green after normal mitochondria is dispersed to the monomeric form. Pretreatment with 20 μM niacin against UV dramatically decreased the green/red fluorescence ratio (P<0.01) in comparison with UV only, and the apoptotic cells dropped from 26.10±4.57% to 18.92±3.26% (P<0.01).

### AKT, TSC2 and mTOR are required for UV-induced AKT cascade activation

We next examined whether the AKT cascade is activated upon UV radiation. The results showed that UV radiation activates the EGFR/AKT/mTOR pathway in a time- and dose-dependent manner. UV radiation (30 mJ/cm^2^) activates AKT at the highest level. The peaks of EGFR/AKT/mTOR activation take place between 30 and 60 min at the UV dose of 30 mJ/cm^2^ (Fig. 2A and B). Previous studies have demonstrated the key role of AKT in mTOR activation in response to growth factors (32). To investigate the role of AKT in UV-induced mTOR/S6 activation, AKT cascade inhibitors were used. The results show that UV does not induce AKT/mTOR/S6 activation in cells treated with the EGFR inhibitor, PD153035, or the AKT inhibitor, LY294002 (Fig. 2D and E), suggesting that both EGFR and AKT are required for UV-induced mTOR/S6 activation. Previous studies have also shown that the regulation of S6K and 4E-BP1 by AKT occurs primarily through the phosphorylation and inactivation of TSC2 at Tyr1462 (34), leading to increased phosphorylation of mTOR and downstream S6K and 4E-BP1. We next examined the role of TSC2 in S6K activation upon UV radiation. As shown in Fig. 2F, UV-induced mTOR/S6 activation is modulated by TSC2. Transfection with TSC2 siRNA specifically silenced TSC2 by approximately 60%, and the downstream mTOR and S6 signals were partially inhibited (Fig. 2F).

### Niacin, in contrast to AKT cascade inhibitors, affects UV-induced apoptosis in HaCaT cells

As demonstrated, niacin protects against UV-induced cell death and cell apoptosis. The AKT cascade activation is induced by UV radiation. Taken together, we conclude that the AKT cascade signal activation serves as a critical upstream signal against UV, serving as a pro-survival signal against UV-induced cell apoptosis. To determine whether the AKT signaling pathway is involved in the pro-survival and anti-apoptotic effects of niacin, cells were treated with AKT cascade kinase inhibitors independently, such as the EGFR inhibitor, PD153035, the AKT inhibitor, LY294002 and the mTOR inhibitor, rapamycin. As previously shown, treatment with PD153035, LY294002 and rapamycin resulted in the increase of UV-induced apoptosis. Living cells were decreased successively from 93.21±2.74% to 80.08±3.20% while the percentages of apoptotic cells were successively increased from 6.35±0.32% in the control to 18.39±0.55% (P<0.01) in the rapamycin group. Independent treatment with LY294002 and rapamycin seemed to affect cells efficiently. The contribution of the AKT cascade signal activation after UV was further detected by pretreating cells with inhibitors before UV exposure. Treatment with LY294002 and rapamycin were found to have less influence on the UV-induced loss of cell viability in the cells in comparison with PD98059. However, LY294002 has a more critical role in the UV effect. The UV-induced apoptosis ratio was 36.71±3.67% compared to others. Last, we treated niacin-treated cells with inhibitors prior to UV. This led to an insignificant decrease of UV-induced cell apoptosis (P>0.05) except for PD98059 which increaed apoptotic cells (P<0.05).

### Niacin protects against UV-induced apoptosis via enhancement of AKT and mTORC/S6 activation

We have shown that niacin pretreatment protects against UV-induced cell death and apoptosis in keratinocytes (HaCaT cells) (Figs. 1 and 2). AKT and the downstream signal mTOR/S6 are important for the protective effect of niacin, so next we examined whether niacin is able to induce AKT/mTOR/S6 activation in HaCaT cells. The results showed that niacin strongly induces AKT and the downstream mTOR/S6 activation at 30 min (Fig. 4A). Furthermore, niacin induces little activation of MAPK (ERK and JNK) compared to the UV group which strongly activates MAPK (p38) (Fig. 4C). We also demonstrated that UV-induced AKT/mTOR/S6 activation serves as a pro-survival signal (Fig. 2). Next we examined the possible role of niacin on UV induced AKT/mTOR/S6 activation. As shown in Fig. 4B, niacin pretreatment largely enhances UV-induced AKT/mTOR/S6 activation in HaCaT cells. The AKT inhibitor, LY294002 largely neutralizes the protective effects of niacin (Fig. 4E) and shows a low mitochondrial membrane potential, indicating that AKT activation is necessary for niacin’s protective effects against UV-induced cell apoptosis.

## Discussion

Despite previous research showing that niacin reduces the immunosuppressive effects of UV both *in vivo* and *in vitro* (35), at least in part by providing energy repletion to UV-irradiated cells for it can normalize subsets of apoptosis and cellular energy loss effects (8,36), the precise molecular mechanisms underlying the cytoprotective and anti-apoptotic effects remain largely unknown. Here, we showed that treatment with niacin led to efficient suppression of UV-induced cell death and apoptosis in keratinocytes (Figs. 1 and 2). We also found that the treatment of niacin could recover the changed mitochondrial membrane potential. These data suggest that niacin can protect against UV-induced mitochondrial dysfunction (Fig. 2). The fact that niacin protects the cells from apoptotic cell damage appears to be applicable to the protection from UV irradiation of keratinocytes, which are the primary cell type in the epidermis and play a key role in the body’s initial line of defense.

To understand the molecular mechanism of the anti-apoptotic effect of niacin in UV-treated keratinocytes, first we analyzed several signaling pathways related to UV-induced apoptosis in HaCaT cells. We found that the short time-dependent regulation of the AKT cascade and MAPK feedback activation is involved in HaCaT cells after UV exposure. AKT is well known to be differentially activated depending on the type of extracellular stimuli. As suggested in previous studies, MAPK/JNK/p38 activation may be essential for UV-induced apoptosis, but the activation of AKT, mTOR, S6 can be the pro-surviving signals against UV-induced apoptosis. Some plant flavonoids with anti-apoptotic properties activate the MAPK/AKT/NF-κB pathway (37–39). We found that niacin pretreatment largely enhances UV-induced AKT/mTOR/S6 activation in HaCaT cells (Fig. 4). Therefore, the PI3K/AKT cascade is considered as the canonical pathway involved in the protection of UV-induced apoptosis followed by EGFR kinase activation. As indicated in the Fig. 3 apoptosis assay, EGFR could relatively strengthen the damage of UV; AKT and mTOR inhibitors could largely neutralize the protective effects of niacin against UV, suggesting that AKT signaling activation is necessary for niacin’s protective effects against UV-induced cell death and apoptosis.

In addition to stimulating cell growth, mTOR also promotes cell survival. eIF4E serves as an important downstream effectors of mTOR in the control of cell survival through the 4E-BP1 (40–46). The translation and expression of mRNAs encoding a few major anti-apoptotic proteins including (XIAP, c-IAP1, Bcl-XL and BCl-2) are mTORC1 and cap-dependent (47). S6K1 is another mTOR target that plays a role in the apoptosis resistance of cancer cells (48–50). Previous studies (51) together with our current work demonstrate that mTOR activation serves as a pro-survival UV-induced cell apoptosis signal (Figs. 2 and 4). AKT, by phosphorylation and inhibition of TSC2, serves as the upstream signal for UV-induced mTORC1 activation (Fig. 2). Importantly, UV-induced TSC2 and S6K phosphorylation were almost abolished by pharmacological inhibitors of AKT (Fig. 2). Taken together, we conclude that AKT by phosphorylating and inhibiting TSC2, acts as an upstream signal for UV-induced mTOR activation, and the latter serves as a pro-survival signal against UV-induced cell death and apoptosis.

Although the PI3K/AKT and its downstream substrate mTOR (S6K and 4E-BP1 phosphorylation, rapamycin sensitive) pathway are well-established, the identity of the kinase responsible for phosphorylating AKT at Ser473 remains elusive until in recent years, when it was revealed to be mTORC2 (46,52–54). mTORC2 is a complex of mLST8, rictor (rapamycin-insensitive companion of mTOR), and mSin1 with mTOR (46,52–56). Aside from AKT hydrophobic motif phosphorylation, mTORC2 has also been implicated in the phosphorylation of the AGC kinase, PKCα (46,57), the regulation of actin cytoskeleton reorganization (46) and development of prostate cancer in PTEN deficient mice (58). Ablation of mTORC2 activity impairs the phosphorylation of only a subset of AKT targets including FoxO1/3a, while leaving other AKT targets such as TSC2 and glycogen synthase kinase 3 (GSK-3) as well as the mTORC1 effectors S6K and 4E-BP1 unaffected (46,57,59).

In conclusion, we found for the first time that niacin pretreatment protects against UV-induced cell death and apoptosis by enhancing the pro-survival pathways including AKT, mTOR and S6 in skin keratinocytes (HaCaT cells). Oral and external niacin and nicotinamide are both safe and inexpensive and appear to be promising chemopreventive supplements for reducing the mutagenic, immunosuppressive and cell damage effects of sunlight (60). To our knowledge, this is also the first study providing a molecular mechanism to support that niacin can be utilized as a skin photodamage protective agent.

## Figures and Tables

**Figure 1:** Niacin protects against UVB induced cell death in HaCaT cells. HaCaT cells were pretreated with niacin (0, 5, 10, 20 and 40 μM) for 1 h, followed by 30 mJ/cm^2^ UV radiation. After incubation at 37°C for 24 h, cell viability was detected by the MTT assay. The values in the figure are expressed as the means ± standard deviation (SD). ^*^P<0.05, ^**^P<0.01 vs. the UV-treated niacin-free group. All experiments were repeated at least three times and similar results were obtained.

**Figure 2:** AKT, TSC2, mTOR and S6 are required for UV-induced AKT cascade activation. (A and B) HaCaT cells were exposed to different dosages of UV radiation (0, 5, 15, 30, 60, 120 mJ/cm^2^) for 30 min and for different durations of 30 mJ/cm^2^ UV respectively. p-EGFR (Tyr1068), p-AKT (Ser473), p-4E-BP1 (Ser65) were detected by western blotting. (C) HaCaT cells were pretreated with 20 μM niacin, followed by UV radiation (0, 15, 30, 60 mJ/cm^2^), then stained with the JC-1 probe and imaged by fluorescent microscope. The individual red and green average fluorescence intensities are expressed as the ratio of green to red fluorescence. An increase on the fluorescence green/red ratio indicates a shift increase in mitochondrial depolarization as an early apoptosis label. HaCaT cells were pre-treated with (D) the EGFR inhibitor, PD153035 (PD, 1 μM); (E) with the PI3K/AKT inhibitor LY294002 (LY, 10 μM) and mTOR inhibitor rapamycin (Rapa, 100 nM), for 1 h, with UV (30 mJ/cm^2^) radiation and cultured for 15, 30 and 60 min. (F) Cells were transfected with Tuberin/TSC2 siRNAII (100 nM) for 48 h prior to UV radiation (30 mJ/cm^2^), for 30 or 60 min. p-EGFR (Tyr1068), p-AKT (Ser473), p-AKT (Thr308), p-TSC2 (Thr1462), p-mTOR (Ser2448), p-S6K (Thr389), p-S6 (Ser235/236), p-4E-BP1 (Ser65) and total AKT antibody were used by western blotting. All experiments were repeated at least three times and similar results were obtained.

**Figure 3:** Niacin protects HaCaT cells from UV-induced apoptosis cooperated with different AKT cascade inhibitors. HaCaTs were pre-treated with 20 μM niacin (NA) for 30 min, and then incubated with different inhibitors for 30 min until 30 mJ/cm^2^ of UV radiation. PD, LY, RaPa are abbreviations for PD153035, LY294002, and rapamycin respectively. Twenty-four hours post-treatment the number and percentage of apoptotic and necrotic cells were quantifled by FACS after cells were washed and stained with Annexin V and PI. Apoptotic cells were determined by counting the percentage of early apoptotic cells Annexin V(+), PI(−) cells plus the percentage of late apoptotic Annexin V(+), PI(+) cells. Normal living cells are presented as Annexin V(−), PI(−), respectively. The values in the figure are shown as mean ± SD of at least three separate experiments. ^*^P<0.05, ^**^P<0.01 vs. the control group; ^#^P<0.05, ^##^P<0.01 vs. the UV only group; and ^&^P<0.05 when comparing the PD+UV and PD+NA+UV group.

**Figure 4:** Niacin protects against UV-induced apoptosis via enhancement of AKT/mTOR/S6 activation. (A) HaCaT cells were treated with niacin (NA, 20 μM) and cultured for 5, 15, 30, 60 and 120 min. p-EGFR (Tyr1068), p-AKT (Ser473), p-mTOR (Ser2448), p-S6K (Thr389), p-S6 (Ser235/236), p-4E-BP1 (Ser65), total AKT and β-actin antibody were used for western blotting. (B and C) HaCaT cells were pretreated with or without niacin (20 μM) for 1 h, followed by UV (30 mJ/cm^2^) radiation and cultured for the indicated time, p-EGFR (Tyr1068), p-AKT (Ser473), p-mTOR (Ser2448), p-S6K (Thr389), p-S6 (Ser235/236), p-4E-BP1 (Ser65), p-p38 (Thr180/Tyr182), p-JNK (Thr183/Tyr185), p-ERK1/2 (Thr202/Tyr204), p38 MAPK, JNK total AKT and β-actin were detected by western blotting. (D) HaCaT cells were pretreated with niacin (20 μM) for 1 h, followed by UV radiation (30 mJ/cm^2^) and cultured for 1 h, p-AKT (Ser473) and p-S6 (Ser235/236) were detected by confocal microscopy. (E) HaCaT cells were pre-treated with niacin and LY294002 separately or in combination, after UV (30 mJ/cm^2^) radiation; mitochondrial depolarization was observed the same way in Fig. 2C.
